# A Robust Context-Based Deep Learning Approach for Highly Imbalanced Hyperspectral Classification

**DOI:** 10.1155/2021/9923491

**Published:** 2021-07-06

**Authors:** Juan F. Ramirez Rochac, Nian Zhang, Lara A. Thompson, Tolessa Deksissa

**Affiliations:** ^1^Department of Computer Science & Information Technology, University of the District of Columbia, Washington, DC 20008, USA; ^2^Department of Electrical & Computer Engineering, University of the District of Columbia, Washington, DC 20008, USA; ^3^Biomedical Engineering Program, Department of Mechanical Engineering, University of the District of Columbia, Washington, DC 20008, USA; ^4^Water Resources Research Institute, University of the District of Columbia, Washington, DC 20008, USA

## Abstract

Hyperspectral imaging is an area of active research with many applications in remote sensing, mineral exploration, and environmental monitoring. Deep learning and, in particular, convolution-based approaches are the current state-of-the-art classification models. However, in the presence of noisy hyperspectral datasets, these deep convolutional neural networks underperform. In this paper, we proposed a feature augmentation approach to increase noise resistance in imbalanced hyperspectral classification. Our method calculates context-based features, and it uses a deep convolutional neuronet (DCN). We tested our proposed approach on the Pavia datasets and compared three models, DCN, PCA + DCN, and our context-based DCN, using the original datasets and the datasets plus noise. Our experimental results show that DCN and PCA + DCN perform well on the original datasets but not on the noisy datasets. Our robust context-based DCN was able to outperform others in the presence of noise and was able to maintain a comparable classification accuracy on clean hyperspectral images.

## 1. Introduction

Advances in data collection and data warehousing technologies have led to a wealth of massive repositories of data. Together with active research in artificial intelligence, big data science promises mountain ranges of unexplored datasets and the smart tools to extract relevant information. An important goal in computer-based hyperspectral imaging is to be able to accurately perform this information mining without human work. Government, industry, and academia sectors seek to automate this process. They find it valuable for their future to be able to reduce the human requirement in core processing tasks, such as segmentation, classification, and its applications.

Ever since Vapnik's [1, 2] work transformed the statistical learning theory community, research has indicated the considerable potential of SVM in supervised classification, However, in many real-world classification problems such as remote sensing, medical diagnosis, object recognition, and business decision-making, the costs of selecting a poor kernel for high dimensional data is too high in terms of computational performance and a handicap to robust, real-time hyperspectral classification and segmentation.

More recently, deep networks have dominated classification problems, such as image segmentation. Convolutional-based neural networks or CNNs are driving advances in recognition. CNNs are not only improving for all domains of image classification [3–7] but also making progress on object detection [8–10], key-point-based prediction [11, 12], and local correspondence [13]. The natural next step in the progression from coarse to fine inference is to make a prediction at every pixel. Prior approaches have used Deep CNNs for image segmentation [14–20], in which each pixel is labeled, but with shortcomings that this work addresses.

Typically, DCN-based algorithms use the output of the last layer of the network to assign category labels. Imposing a softmax layer on top of a fully-connected dense layer, DCN focuses on semantic information. However, when the task we are interested in is more granular, such as one of classifying mixed pixels or dealing with imbalanced multiclass classification of hyperspectral images, these last layers are not optimal.

Image segmentation faces yet another challenging gap: global information answers the what, while local information provides the where. It is not immediately clear that deep convolutional neural networks for image classification yield a structure sound enough for accurate, pixel-wise multiclass classification. Moreover, when working with high dimensional features, there is often no go-to algorithm that is exact and has acceptable performance. To obtain a speed improvement, many practical applications are forced to settle for approximation approaches, in which they do not return exact answers. In practice, numerical optimizations and fast approximation saturate the spectrum of algorithms and research. However, image segmentation can also be explored as the reconstruction to a low-quality image from its high quality observations. This point of view has many important applications, such as low-level image processing, remote sensing, medical imaging, and surveillance.

There are also paramount applications that would benefit from advances in unsupervised image segmentation, such as medical applications and homeland security. Early detection of tumors, kidney disease, heart disease, microbleeds, and microdamages is critical to worldwide public health. There is significant research and new investments for advancing magnetic resonance imaging technology that can accurately aid in early diagnosis. The authors in [21] reviewed the principles and applications of a gradient echo MRI, the so called *T*2∗ weighted. During COVID, the pharmaceutical industry joins forces with academia to develop algorithms for automated assessment of large-scale datasets [22]. Detection of illicit drugs, warfare agents, and dangerous substances is critical to security. The authors in [23] introduced a new technology that can rapidly detect explosives using a thermal imager. This thermal spectroscopy pushes the boundaries of traditional image and signal processing techniques.

The problem is that the state-of-the-art in machine learning and data science demands for abundance of labeled samples, which require domain expert input. This is not feasible to spend time and effort labeling training samples. It is more efficient to develop a new method that scales and requires small number of labeled training samples.

Moreover, noise is a challenging variable, specially within imbalanced data. Hyperspectral imaging is such a data containing highly-imbalanced classes. Multiclass classification using DCN suffers from the presence of noise. Therefore, this study proposes a method that can address these challenges using a deep learning-based image clustering model that combines both an adaptive dimensionality reduction approach and a robust feature augmentation approach which can cluster different types of imaging datasets with high positive predictive value.

The main contribution of this paper is a new preprocessing approach to deal with noisy, highly-imbalanced hyperspectral classification. In Section 2, we present a literature review. In Section 3, we explain our approach. In Section 4, we explain our experiments, while in Section 5, we compare our results. And in Section 6, we present our conclusions and future lines of research.

## 2. Related Works

This section presents previous works and relevant literature in the areas of dimensionality reduction, feature augmentation, noise reduction, and hyperspectral image classification.

### 2.1. Dimensionality Reduction

As big data, cloud computing becomes the standard for data storage, and high dimensional datasets are more and more commonplace. To process such large oceans of data, dimensionality reduction offers two options: feature projection and feature selection. Feature projection techniques transform data from a highly dimensional space to a new space with a lower dimensionality. Principal Component Analysis is one of the most popular linear transformations. In [24] the authors effectively conducted a dimension reduction by applying the principal component analysis to highly overlapped photo-thermal infrared imaging dataset. Feature selection techniques are an alternative that aims to choose the most information-rich features and discard irrelevant features and noise. The authors in [25, 26] present different feature selection techniques to integrate spectral band selection and hyperspectral image classification in an adaptive fashion, with the ultimate goal of improving the analysis and interpretation of hyperspectral imaging.

Recent literature [27] proposes a Kronecker-decomposable component analysis model that combines dictionary learning and component analysis with great results on low rank modeling. The Kronecker product is compatible with the most common matrix decomposition. Therefore, it can be used to learn low-ranking dictionaries in tensor factorization. It also can effectively remove noise.

Principal Component Analysis [28] or PCA is a classical dimensionality reduction with multiple implementations. One intuitive implementation consists of six steps: standardization, covariance, eigenvalues, eigenvectors, reduction, and projection. This formulation is based on maximizing variance within a low-dimensional projection. There are other formulations that scale better to high dimensionality. One of such solver implementations consists of breaking down PCA into two easy-to-calculate subproblems: alternating least square linear regressions [29] using an iterative algorithm based on the idea that the product of principal orthogonal components can be an approximation to the original data.

Despite the fact that PCA is among the most established techniques for dimensionality reduction, the story does not end here. There are many other techniques that show great empirical applications and theoretical guarantees. The authors in [30] introduced a Forward Selection Component Analysis and obtained comparable results to PCA and Sparse PCA. And in [31, 32], anomaly and change detection was carried out with great success in hyperspectral imaging. Yet, [33] suggests PCA as yet a powerful preprocessing step to denoise data. Similarly to numerous other noise reduction methods including patents [34], PCA works under the assumption that the signal needs to be cleaned from the same global noise.

### 2.2. Image Classification

Deep learning and big data science are the state-of-the-art in image classification. From support vector machines to convolutional neural networks to spectral clustering, both academia and industry keep pushing for more innovative research. Collaborative and in particular interdisciplinary research is needed to bring these advances to other fields and transform innovations into applications. The authors in [35] and [36] bear witness to the benefits of incorporating diversity to research teams. With authors with top degrees in civil engineering, computer science, and communications and graduate and undergraduate authors, these teams show that in order to push the science forward we need the help of everyone.

There are many classic image segmentation algorithms, from simple thresholding to similarity-based clustering to connectedness and discontinuity-based detection. Threshold-based image segmentation seeks to divide the scale range into background and a set of target foregrounds based on global or local information, for instance, minimizing their interclass variance, maximizing entropy, and/or fuzzy sets theory. One big advantage of using these simple methods is the low computational cost in terms of code complexity which is evident in fast speed operation. This is mainly because thresholding does not take into account spatial information. One drawback is that in the presence of noise, results are not optimal. Similarity-based segmentation uses the idea of clustering based on certain aggregation in feature space. K-means clustering is one of the most well-known unsupervised algorithms. K-means groups together pixels based on their distance; hence, it is considered a distance-based partition method. Connectedness-based image segmentation is a region growing approach that links together points with similar features creating homogeneous and smoothly-connected segments. Discontinuity-based image segmentation seeks to detect object edges or high changes in intensity. Its motivation comes from the idea that there is always a discontinuity between different regions or segments. These discontinuities can be detected using derivatives. Prewiit, Sobel, and Laplacian operators are among the most popular differential operators for spatial domain edge detection which can be applied using convolution for image segmentation.

There are also emerging machine learning and deep learning approaches. Support Vector Machines or SVM is a machine learning algorithm that models classification tasks as optimization problems subject to inequality constraints. The original algorithm [1] was invented by Vapnik and Chervonenkis in 1963. SVM uses a dual Lagrangian, which depends only on labeled samples. The traditional SVM philosophy consists of finding the hyperplane that maximizes the margin between points of different classes. Note that the hyperplane is at the centre of the margin that separates the two classes. The kernel trick was introduced in [2] by Cortes in 1995. This hyperplane is denoted by the perpendicular vector *w* from the origin and it is characterized by (12). Introduce a new variable Y subscript *i*-th such that *Y*_i_ is positive (+1) for gray samples and it is negative (–l) for yellow samples. This optimization problem is solved using a Lagrangian multiplier (13). After applying the partial derivatives, it is evident that the solution only depends on the inner product of the supporting vectors ***x***_***i***_. Different kernel functions SVM may be employed to solve nonlinearly separable samples. Thus, SVM performs so well on binary classification.

Deep Convolutional Neuronets or DCN is a deep learning algorithm that models a classification task as series of convolutional layers, pooling layers, dropout, and an activation layer usually consisting of a softmax function. CNN-based learning has recently achieved expert level performance in various applications. In [37] the authors present a deep fully convolutional neural network for semantic pixel-wise segmentation. Evaluation of the decoder variants shows that accuracy increases for larger decoders for a given encoder network. Experimental results on road scenes and indoor scenes show that the proposed SegNet outperforms other segmentation benchmarks.

Some other applications of DCN-based segmentation are listed in [38, 39] and [40]. In [38], the authors extended the original DeepLab with more speed, accuracy, and simplicity by compiling a comprehensive evaluation on benchmark and challenging datasets, such as PASCAL VOC 2012, Cityscapes, among others. In [39] the authors present a new unsupervised image segmentation based on the centre of a local region. The authors validated their work on 2D and 3D medical images. MATLAB was used to implement the approach on X-rays, abdominal and cardiovascular MRI images. In [40] the authors present an image segmentation approach that recasts the problem into a binary pairwise classification of pixels.

Deep learning high speed and accuracy come with a price: subject matter expert labor to label. DCN-based approaches are supervised learning and labeled samples are needed in abundance which results in a high demand for SME input. Despite the shortcomings, multiple research initiatives are pushing the boundaries of noninvasive medicine, remote sensing, and natural language processing. Deep learning-based models stand at the core of these emerging applications.

### 2.3. Applications in Medical Image Processing

U-NET deep FCN structure is highly applicable for medical image segmentation. Multiple U-NET variants [41–43] and domain specific models [44] have been applied to process medical images. For instance, [41] presents a U-Net variant for image segmentation on brain tumor MRI scans while [42] presents another U-Net variant based on nested and dense skip connections for medical image segmentation. Moreover, [43] introduces a robust self-adapting U-Net-based framework for medical image segmentation. And [44] adds the emerging attention mechanism to a nested U-Net architecture for image segmentation on liver CT scans. One interesting medical application of image segmentation using a deep learning model is presented in [45]. A new hybrid of the classic V-Net architecture is used to help detect kidney and renal tumors on CT imaging with successful performance of medical segmentation. This wealth of deep learning research branches out from the U-Net model and provides expert-level solutions to medical image segmentation.

Recently, one shot learning models have been proposed to detect COVID-19 using medical images. Signoroni et al. [46] introduced a learning-based solution designed to assess the severity of COVID-19 disease by means of automated X-ray image processing, a domain specific implementation of [42]. Furthermore, [47] compiles an early survey of medical imaging research toward COVID-19 detection, diagnosis, and follow-up. One of their findings is the proliferation of AI-empowered applications which use X-rays and/or CT scans to provide partial information about patients with COVID-19. This reinforces the sense that deep learning-based solutions are widely used in medial image processing.

Tensor-based learning has also been incorporated into medical image processing and hyperspectral imaging. An et al. [48] presented a tensor-based low rank decomposition model for hyperspectral images and evaluates its classification accuracy on hyperspectral cubes. Moreover, the authors in [49] proposed another tensor-based representation to better preserve the spatial and spectral information and capture the local and global structures of hyperspectral images. Yet these models do not focus on imbalanced datasets nor try to solve the denoising problem. Recently, in the field of optical coherence tomography (OCT) [50] has introduced a tensor-based learning model, which tackles the denoising problem on high resolution OCT medical images with great results. However, it is unclear how well tensor-based models would represent the structure of imbalance datasets and will remain outside the scope of our work.

### 2.4. Applications in Natural Language Processing

Natural language processing (NLP) is a field with multiple-machine-learning- (ML-) and deep-learning- (DL-) based research initiatives. With sentiment analysis as a fundamental task of NLP, researchers have proposed several domain specific applications of ML- and DL-based frameworks. The main challenge encountered in machine-learning-based sentiment classification is the unmanageable amount of data. To address this challenge, [51] presents an ensemble learning (EL) approach for feature selection, which successfully aggregates several different feature selection results, so that we can obtain a more robust and efficient feature subset. Moreover, [52] also explores the predictive performance of different feature engineering schemes, four supervised ML-based algorithms and three EL-based methods obtaining experimental results that yield higher predictive performance compared to the individual feature sets. Furthermore, in [53], the author presents yet another comprehensive analysis this time of keyword extraction approaches with empirical results that indicate an enhanced predictive performance and scalability of keyword-based representation of text documents in conjunction with EL-based models.

Sentiment analysis is a critical task of extracting subjective information from online text documents, mainly based on feature engineering to build efficient sentiment classifiers. To improve the feature selection process, [54] proposes and validates the effectiveness of a hybrid ensemble pruning scheme based on clustering and randomized search for text sentiment classification. Sentiment analysis can be reduced to a text classification problem. However, the text classification problem suffers from the curse of high dimensional feature space and feature sparsity problems. To mitigate and lift this curse, [55] explores several classification algorithms and EL-based methods on different datasets.

To recognize sentiment in information-rich but unstructured text, [56] presents a DL-based approach to sentiment analysis on product reviews with outperforming results. Since Twitter can serve as an essential source for several applications, including event detection, news recommendation, and crisis management, in [57], the author presents a DL-based scheme for sentiment analysis on Twitter messages with consistent and encouraging results.

ML- and DL-based models are at the core of NLP research. For instance, Onan [58] indicated that DL‐based methods outperform EL-based methods and supervised ML-based methods for the task of sentiment analysis on educational data mining. And the list does not stop here. Onan [59] indicated that topic-enriched word embedding schemes utilized in conjunction with conventional feature sets can yield promising results for sarcasm identification. Onan [60] presented first usage of supervised clustering to obtain diverse ensemble for text classification and compare it to ML- and DL-based models. Onan and Toçoğlu [61] employed a three-layer stacked bidirectional long short-term memory architecture to identify sarcastic text documents with promising classification accuracy results. Onan [62] presented an extensive comparative analysis of different feature engineering schemes and five different ML-based learners in conjunction with EL-based methods.

## 3. Methodology

The main objective of our proposed approach is to optimize the performance of DCN on hyperspectral images. We developed a context-based feature augmentation approach to provide resistance against noise to deep learning classification of highly imbalanced hyperspectral images. The classification apparatus used in this study relies on a deep convolutional neuronet (DCN) to perform multiclass classification based on findings in [63]. The input to this network is a highly imbalanced hyperspectral image or cube.  Figure 1 shows a hyperspectral cube.  Figure 2 shows a 1-by-1 column along the spectral dimension.

Our proposed approach will be a preprocessing module in this classification apparatus as shown in Figure 3. Our four-step approach is introduced as follows. Full details are presented in Sections 3.1through 3.2.

- Local gradients are *feature vectors* of differences, defined in Section 3.1. In this step, we calculate these *feature vectors* for each pixel *p* in the hyperspectral cube, as differences between the pivotal pixel *p* and its surrounding pixels in a 3-by-3-by-3 *local neighborhood.* This set of differences will constitute the *local gradients* of *p.*
- Reference clusters are *feature vectors* of high and low thresholds, defined in Section 3.2. In this step, we calculate these *feature vectors* for each pixel *p* in the hyperspectral cube, as statistical thresholds of the surrounding 9-by-9 *reference neighborhood.* This set of thresholds will constitute the *reference clusters* of *p.*
- Prototype contexts are *feature vectors* of similarity, defined in Section 3.3. In this step, we calculate these *feature vectors* for each pixel *p* in the hyperspectral cube, as the degree of membership of the *local gradients* to the *reference clusters.* This set of similarity degrees will constitute the *prototype contexts* of *p.*
- Concatenated features are all *feature vectors*, defined in Sections 3.1 and 3.2. In this step, we concatenate *local gradients*, *reference clusters,* and *prototype contexts* into one context-based *feature vector* for each pixel *p* in the hyperspectral cube.

### 3.1. Calculate Local Gradients

The first step of our approach is to calculate the *local gradients* [64].  Figure 4 shows a pivotal pixel *p*(1, 1, 1) in its 3-by-3-by-3 *local neighborhood*. The *local gradient ****χ*** is the set of gradient differences {*d*_1_, *d*_2_, *d*_3_,…, *d*_13_}, where *d*_i_ is the magnitude of the differences between *p* and its direct neighbors for each discrete direction *i*. For instance, in direction *i* = 1, *d*_1_ is equal to |*p*_1,1,1_ − *p*_2,1,1_| + |*p*_1,1,1_ − *p*_0,1,1_|, whereas, in direction *i* = 10, *d*_10_ is equal to |*p*_1,1,1_ − *p*_2,2,2_| + |*p*_1,1,1_ − *p*_0,0,0_|. Such *local gradients* are calculated for each pixel *p*_*i,j,k*_ within the hyperspectral cube.

It is important to note that this moving cubic-shaped *local neighborhood* only uses partial data around the borders of the hyperspectral image. Thus the indexes, i, j, k, will only run from 1 to the dimension length −1 for each dimension *x*, *y*, *z*.

### 3.2. Calculate Reference Clusters

The second step of our approach is to calculate the *reference clusters* [64].  Figure 5 shows a pivotal pixel *p*(5, 5, 5) in its 9-by-9 *reference neighborhood*. The *reference clusters ****ζ*** is the sets of high and low thresholds {hi_1_, hi_2_, hi_3_,…, hi_13_}, {lo_1_, lo_2_, lo_3_,…, lo_13_}, where hi_i_ is the central value of the high-valued gradients and lo_i_ is the central value of the low-valued gradients within *p'*s *reference neighbors* for each discrete direction *i*. We calculate these central values using the mean*μ* and variance *σ*^2^ equations presented in (1) and (2) to set hi = *μ*+2*σ* and lo = *μ*–2*σ*. Such *reference clusters* are calculated for each pixel *p*_*i,j,k*_ within the hyperspectral cube.

(1) $$\begin{array}{c} \mu_{i,j,k,d}=\frac{1}{N\times M}\sum_{n=0}^{N-1}\sum_{m=0}^{M-1}x_{i+n,i+m,k,d}, \end{array}$$

(2) $$\begin{array}{c} \sigma^{2}=\frac{1}{N\times M}\sum_{n=0}^{N-1}\sum_{m=0}^{M-1}{\left(x_{i+n,i+m,k,d}-\mu_{i,j,k,d}\right)}^{2}. \end{array}$$

It is important to note that this moving square-shaped *reference neighborhood* only uses partial data around the borders of the hyperspectral image. Thus the indexes, *i*, *j* will only run from 5 to the dimension length −5 for each spatial dimensions. It will use however all the spectral bands on the *z* dimension.

### 3.3. Construct Prototype Contexts

The third step of our approach is to construct the *prototype contexts*. The *prototype contexts ****κ*** is the sets of similarity features {*c*_1_, *c*_2_, *c*_3_,…, *c*_13_} where *c*_i_ is the *prototype context* with the highest degree of membership for each discrete direction *i*. We calculate this degree of membership *M* with the equation presented in (3)–(6) where *D*^2^ is the square of the Mahalanobis distance, *χ* is the vector of local gradients, *κ* is the vector of prototype contexts, *W* is the inverse pooled covariance matrix, and the *K* factor is equal to the square root of the product between the highest value in *χ* and the highest value in *κ*. Such *prototype contexts* are calculated for each pixel *p*_*i*,*j*,*k*_ within the hyperspectral cube.

(3) $$\begin{array}{c} M\left(\chi \right)=\max\left(0,\;1-\frac{D}{\sqrt{K}}\right), \end{array}$$

(4) $$\begin{array}{c} D^{2}\left(\chi ,\kappa \right)={\left(\chi -\kappa \right)}^{T}W^{-1}\left(\chi -\kappa \right), \end{array}$$

(5) $$\begin{array}{c} W\left(\chi ,\kappa \right)=\frac{1}{2}\mathrm{cov}\left(\chi \right)+\frac{1}{2}\mathrm{cov}\left(\kappa \right), \end{array}$$

(6) $$\begin{array}{c} K\left(\chi ,\kappa \right)=\max\left(\chi \right)\times \max\left(\kappa \right). \end{array}$$

### 3.4. Concatenated Augmented Features

The fourth step of our approach is to concatenate all *features vectors*. These *feature vectors* consist of the *local gradients*, *reference clusters*, and *prototypes contexts*. Such *context-based feature vectors* are concatenated for each pixel *p*_*i*,*j*,*k*_ within the hyperspectral cube.

Figure 6 shows how our context-based approach integrates into a deep learning classification model. Note that to evaluate the robustness of our approach, we added a synthetic noise to the original datasets. This noise was generated using a Gaussian equation. And classification accuracy was used as the main measurement to compare the performance of the model and in particular the resistance to noise in imbalanced hyperspectral images. Details are presented in the following section.

## 4. Experiments

In this section, we describe the datasets, dataset partition policy, and experimental settings. Multiple settings are designed to evaluate the performance of our approach on noisy and clean data, as well as on imbalanced and balanced data.

### 4.1. Datasets

Four datasets were used in our experiments. The first two are the Pavia Centre and Pavia University datasets. These two datasets were acquired by the ROSIS sensor during a flight campaign over Pavia, Italy. The original Pavia Centre dataset is a hyperspectral cube with a spatial resolution of 1096 × 715 and 102 spectral bands, and the original Pavia University dataset is a hyperspectral cube with a spatial resolution of 610 × 340 spatial pixels and 103 spectral bands. The corresponding ground truths differentiate nine classes. For more details, please visit the following link. This link was last accessed on February 1, 2021 (http://www.ehu.eus/ccwintco/index.php/Hyperspectral_Remote_Sensing_Scenes#Pavia_Centre_and_University).

It is important to note that the Pavia Centre data are considered a balanced hyperspectral cube, whereas the Pavia University data are considered an imbalanced hyperspectral cube. It is clear from Figure 7 that the Pavia Centre samples are evenly distributed between classes. But, in Figure 8, the majority of Pavia University samples belong to one single class, namely the class *Meadows.* Thus, this predominant class dwarfs minority classes, such as *Shadows*, *Bitumen,* and *Painted Metal Sheets*. This disparity is what makes Pavia University data imbalanced.

To evaluate the robustness of our approach, we added a synthetic noise to the original “*clean*” datasets and produced two additional synthetic datasets. Thus, together with the two clean datasets, two noisy datasets were used in our experiments, corresponding to the noisy Pavia Centre and the noisy Pavia University datasets. Identically to their clean counterparts, the noisy Pavia Centre dataset is a hyperspectral cube with a spatial resolution of 1096 × 715 pixels, 102 spectral bands and 9 distinct classes, and the noisy Pavia University dataset is a hyperspectral cube with a spatial resolution of 610 × 340 pixels, 103 spectral bands and 9 distinct classes.

To produce these noisy datasets, an intermittent irregular noise was incorporated. Equations (7)–(9) were used to generate a noise signal corresponding to a signal-to-noise value of SNR_dB_=120. In (7), *G* and *F* are random variables and *N* follows a Gaussian distribution with a probability density function presented in (8). Similarly to [65], this weighted random noise will follow a Gaussian normal distribution *N*(*μ*, *σ*), where the mean *µ* is zero and the variance *σ* is determined from the signal-to-noise ratio (SNR_dB_) formula presented in (9).

(7) $$\begin{array}{c} G\left(a,b\right)\leftarrow F{\left(m,n\right)}^{\;}+N\left(\mu ,\sigma \right), \end{array}$$

(8) $$\begin{array}{c} N\left(x|\mu ,\sigma^{2}\right)=\frac{1}{\sqrt{2\pi \sigma^{2}}}\exp\left[-\frac{{\left(x-\mu \right)}^{2}}{2\sigma^{2}}\right], \end{array}$$

(9) $$\begin{array}{c} SNR_{dB}=20log_{10}\frac{\mu_{signal}}{\sigma_{noise}}. \end{array}$$

### 4.2. Dataset Partition Policy

Datasets were divided into training and testing sets; 80% of the data was used during the training (a.k.a. model-fitting) phase while the remaining 20% of the data was used for testing (a.k.a. model-prediction) phase. One-fourth of the training set was used as validation set during the fitting phase.  Figure 9 shows the full-partition schema.

To rank our context-based DCN approach, two additional models are implemented: (i) a baseline deep learning approach, namely, DCN, and (ii) a benchmark approach, that is PCA + DCN. And classification metrics are used to evaluate and compare the performance and effectiveness of our approach.

### 4.3. Baseline Experiments

As a baseline, we observe the performance of a deep learning model without any preprocessing on the different hyperspectral datasets. Four types of experiments are included in this section. First, we work on clean data, running individual experiments for balanced and imbalanced datasets. Then, we focus on noisy data, and again we run individual experiments for balanced and imbalanced datasets.

A Deep Convolutional Neuronet (DCN) was used as a baseline to perform the classification. We used a DCN which consists of three types of layers, namely, input layer, hidden convolutional layer(s), and output layer. In Figure 10, the input dataset is shown as a cube. Similarly to [40], the hidden convolutional layers are shown as flat squares, the max-pooling layers in whiter color, and the dropout layer in pale. Straight lines are used to depict fully-connected layers or dense layers. Finally, for multiclass classification, the activation function is based on a softmax function.

During the model-fitting phase, we run for 20 epochs. At this point, the network achieves stability without running into overfitting. DCN used the two original datasets and the two noisy datasets. The results of our fitting phase are presented in Figures 11to 14. The average classification accuracy on clean test data was 86.1 ± 3.9 percent, whereas in noisy data was 66.9 ± 2.9 percent. These results suggest an adversary effect of noise on our basic model.

### 4.4. Benchmark Experiments

As a benchmark comparison, we observe the performance of a deep learning model with noise reduction model as a preprocessing on the different hyperspectral datasets. Similarly, to the previous section, this section presents four types of experiments. First, we work on clean data, running individual experiments for balanced and imbalanced datasets. Then, we focus on noisy data, and again we run individual experiments for balanced and imbalanced datasets.

Principal Component Analysis (PCA) together with DCN was used as a benchmark to perform the classification. Ten principal components are sufficient to represent 99% variability of the data.  Figure 15 shows the Scree Curves for both the Pavia Centre dataset in Figure 15(a) and the Pavia University dataset in Figure 15(b).

As suggested by the Scree Curves, PCA + DCN was implemented using only the first ten principal components. Twenty epochs were used during the model-fitting phase, a.k.a. training phase. In our experimental runs, the dataset partition policy was maintained the same and both the original datasets and the noisy datasets were randomly selected into training, validation, and testing sets.

The results of our fitting phase are presented in Figures 16to 19. The average classification accuracy on clean test data was 84.1 ± 6.1 percent, whereas on noisy data was 37.3 ± 4.7 percent. Compared to the results for vanilla DCN, these results strongly suggest an adversary effect of noise on the principal component-based model. Another important point to analyze is that during training of PCA + DCN on noisy data, the model suffered from overfitting after the 4 epochs as shown in Figure 18.

### 4.5. Enhanced Experiments

We integrate our context-based feature augmentation module as a preprocessing step to the deep learning model. We observe the performance of a context-based deep learning model on the original highly imbalanced hyperspectral dataset. Then, we observe the performance of our enhanced model in the presence of noise. We also run our context-based DCN for 20 epochs using the two original datasets and the two noisy datasets. All context-based features were used to achieve better noise resistance.

The results of the model-fitting phase are presented in Figures 20to 23. The average classification accuracy on clean test data was 87.5 ± 3.4 percent, whereas on noisy data was 85.0 ± 4.2 percent. Compared to previous results, these percentages suggest that our proposed approach exhibits a high-level of accuracy on clean data and robustness against noise on both the Pavia University and the Pavia Centre datasets.

## 5. Results and Discussion

### 5.1. Performance Metrics

Receiver operating characteristic (ROC) curves are used to provide a graphical summary of the performance of our classification model. In this Cartesian plane graph, the *x*-axis denotes the False Positive Rate and the *y*-axis denotes the True Positive Rate. Thus, ROC curves depict False Positive Rate vs. True Positive Rate, where we have the following:

- True Positive Rate is equal to True Positives (TP) divided by the addition of True Positives (TP) and False Negatives (FN), that is, TP/(TP + FN)
- False Positive Rate is equal to False Positives (FP) divided by the addition of False Positives (FP) and True Negatives (TN), that is, FP/(FP + TN)

Precision-Recall (PR) curves provide another graphical tool to evaluate performance of a classification model. In this Cartesian plane graph, the *x*-axis denotes the Recall and the *y*-axis denotes the Precision. Thus, PR curves depict Recall vs. Precision, where we have the following:

- Recall is equal to True Positives (TP) divided by the addition of True Positives (TP) and False Negatives (FN), that is, TP/(TP + FN)
- Precision is equal to True Positives (TP) divided by the addition of True Positives (TP) and False Positives (FP), that is, TP/(TP + FP)

Finally, to compare the performance of each model dataset side by side, we compile a table using the ROC Area under Curve (AUC) Score for each model dataset. To this end, we used the following metrics:

- Accuracy is equal to the quotation between the addition of True Positives and True Negatives divided by the Total Population, that is, (TP + TN)/(TP + TN + FP + FN)
- *F*1-score is equal to two times Precision (*P*) times Recall (*R*) divided by the addition of Precision (*P*) and Recall (*R*), that is, 2*PR*/(*P* + *R*)

### 5.2. Prediction Results

The following detail the classification results during the model-prediction phase. The following present the weighted averages for all performance metrics. First, Tables 1 and 2 present the classification results on the original, “clean datasets”, Pavia Centre and Pavia University, correspondingly. Then, Tables 3 and 4 present the classification results on the synthetic, “noisy datasets”, Pavia Centre with noise and Pavia University with noise, correspondingly.

Our experimental results suggest that all models suffer in the presence of noise, but the negative impact of noise can be mitigated with our proposed context-based approach. Tables 3 and 4 present the precision, recall, F1-score, and overall accuracy scores for DCN, PCA + DCN and our context-based DCN.  Table 3 focuses on the noisy Pavia Centre dataset, while Table 4 focuses on the noisy Pavia University dataset. In both tables, we can observe that our proposed model achieves better results.

### 5.3. Tabular Summary and Analysis

Comprehensive summary tables are presented as follows. A total of three approaches were analyzed: a basic DCN with no preprocessing, a PCA + DCN, and a context-based DCN. They are listed on different rows. Four datasets were used: two without noise referenced as “*clean data*” and the same ones with random noise referenced as “*noisy data*”. Imbalanced datasets are listed on shaded columns of the tables. The values in each cell represent overall classification accuracy.  Table 5 summarizes the overall accuracy of each model during the fitting/learning phase, whereas Table 6 summarizes the overall accuracy of each model during the testing/prediction phase.

It is important to note that during training on labeled samples as well as during testing on new samples, our proposed context-based DCN outperformed both DCN and PCA + DCN, especially in the presence of random noise. PCA + DCN did not perform well for noisy cases because it was not able to remove our synthetic noise signal, which was not just random but also intermittent and irregular.

## 6. Conclusions

Hyperspectral imaging is an area of active research. Deep learning-based approaches to classification are the current state-of-the-art. However, our experimental results showed that in the presence of noisy hyperspectral datasets, these expert-level models underperform. To address this shortcoming, this paper presented a context-based feature augmentation approach to increase noise resistance in highly-imbalanced hyperspectral classification.

On noisy datasets, our robust approach outperformed a basic deep learning model and outclassed a combination of PCA and DCN approach. In addition, on highly-imbalanced noisy data, our context-based DCN approach suffered significant loss in terms of classification accuracy (less than 10%), whereas DCN and PCA + DCN suffered from an alarming 25% and 50% cuts in classification accuracy respectively.

Future lines of research should focus on applying our context-based approach to other noisy datasets in areas such as MRI and other highly imbalanced 3D medical images.

## Figures and Tables

**Figure 1:** A hyperspectral image, where *x* and *y* are spatial dimensions and *z* is the spectral dimension.

**Figure 2:** A hyperspectral column, where *z* is the spectral dimension.

**Figure 3:** Overview of our deep learning hyperspectral classification apparatus.

**Figure 4:** Pivotal pixel *p* inside its local neighborhood.

**Figure 5:** Pivotal pixel *p* inside its reference neighborhood.

**Figure 6:** Overview of our approach as a preprocessing module.

**Figure 7:** Class distribution for Pavia Centre. This dataset is considered balanced because for each class, there is relatively the same number of samples.

**Figure 8:** Class distribution for Pavia University. This dataset is considered imbalanced because for each class, there is not the same number of samples.

**Figure 9:** Partition policy: datasets are divided into 3 parts (20%, 20%, and 60%). The training task uses 60% of the samples. The validation task uses 20%. The testing task uses the remaining 20%.

**Figure 10:** Overview of our deep convolutional neural network.

**Figure 11:** DCNN accuracy and loss during the model-fitting phase using the original Pavia Centre dataset.

**Figure 12:** DCNN accuracy and loss during the model-fitting phase using the original Pavia University dataset.

**Figure 13:** DCNN accuracy and loss during the model-fitting phase using the noisy Pavia Centre dataset.

**Figure 14:** DCNN accuracy and loss during the model-fitting phase using the noisy Pavia University dataset.

**Figure 15:** Scree curves for the (a) Pavia University dataset and (b) Pavia Centre dataset.

**Figure 16:** PCA + DCNN accuracy and loss during the model-fitting phase using the original Pavia Centre dataset.

**Figure 17:** PCA + DCNN accuracy and loss during the model-fitting phase using the original Pavia University dataset.

**Figure 18:** PCA + DCNN accuracy and loss during the model-fitting phase using the noisy Pavia Centre dataset.

**Figure 19:** PCA + DCNN accuracy and loss during the model-fitting phase using the noisy Pavia University dataset.

**Figure 20:** Context-based DCNN accuracy and loss during the model-fitting phase using the original Pavia Centre dataset.

**Figure 21:** Context-based DCNN accuracy and loss during the model-fitting phase using the original Pavia University dataset.

**Figure 22:** Context-based DCNN accuracy and loss during the model-fitting phase using the noisy Pavia Centre dataset.

**Figure 23:** Context-based DCNN accuracy and loss during the model-fitting phase using the noisy Pavia University dataset.

**Table 1:** Model comparison based on prediction results using the original Pavia Centre dataset.

Models	Precision (%)	Recall (%)	*F*1-score (%)	Accuracy (%)
DCN	86.70	89.15	85.11	88.92
PCA + DCN	79.71	88.72	83.82	88.52
Context-based DCN	88.35	89.95	88.05	89.88

**Table 2:** Model comparison based on prediction results using the original Pavia University dataset.

Models	Precision (%)	Recall (%)	*F*1-score (%)	Accuracy (%)
DCN	83.99	83.16	83.08	84.28
PCA + DCN	80.68	79.89	78.37	81.29
Context-based DCN	86.37	85.00	85.50	85.78

**Table 3:** Model comparison based on prediction results using the noisy Pavia Centre dataset.

Models	Precision (%)	Recall (%)	*F*1-score (%)	Accuracy (%)
DCN	85.97	65.14	69.00	68.98
PCA + DCN	84.70	34.10	37.26	40.62
Context-based DCN	86.37	82.14	83.40	88.01

**Table 4:** Model comparison based on prediction results using the noisy Pavia University dataset.

Models	Precision (%)	Recall (%)	*F*1-score (%)	Accuracy (%)
DCN	89.72	67.81	73.22	64.79
PCA + DCN	89.45	40.86	46.02	33.93
Context-based DCN	89.48	88.59	88.50	81.99

**Table 5:** Highest validation accuracy during the training phase (model-fitting).

Models	Clean datasets		Noisy datasets	
	Pavia Centre (%)	Pavia University (%)	Pavia Centre w/noise (%)	Pavia University w/noise (%)
DCN	88.93	84.28	96.44	96.00
PCA + DCN	88.69	81.29	88.66	86.24
Context-based DCN	89.92	85.78	98.22	97.83

**Table 6:** Average accuracy score during the testing phase (model-prediction).

Models	Clean datasets		Noisy datasets	
	Pavia Centre (%)	Pavia University (%)	Pavia Centre w/noise (%)	Pavia University w/noise (%)
DCN	88.92	83.37	68.98	64.79
PCA + DCN	88.52	79.76	40.62	33.93
Context-based DCN	89.88	85.02	88.01	81.99

## Data Availability

The datasets used to support the findings of this study are available at http://www.ehu.eus/ccwintco/index.php/Hyperspectral_Remote_Sensing_Scenes.

## References

[1] Vapnik V. N., Chervonenkis A. Y. (1964). On a perceptron class. *Automation and Remote Control*.

[2] Cortes C., Vapnik V. (1995). Support-vector networks. *Machine Learning*.

[3] Ramirez Rochac J. F., Thompson L., Zhang N., Oladunni T. A data augmentation-assisted deep learning model for high dimensional and highly imbalanced hyperspectral imaging data.

[4] Simonyan K., Zisserman A. Very deep convolutional networks for large-scale image recognition.

[5] Szegedy C., Liu W., Jia Y., Sermanet P. Going deeper with convolutions.

[6] Sermanet P., Eigen D., Zhang X., Mathieu M., Fergus R., LeCun Y. OverFeat: integrated recognition, localization and detection using convolutional networks.

[7] Ramirez Rochac J. F., Liang L., Zhang N., Oladunni T. A Gaussian data augmentation technique on highly dimensional, limited labeled data for multiclass classification using deep learning.

[8] Girshick R., Donahue J., Darrell T., Malik J. (2015). Region-based convolutional networks for accurate object detection and segmentation. *IEEE TPAMI.*.

[9] He K., Zhang X., Ren S., Sun J. Spatial pyramid pooling in deep convolutional networks for visual recognition.

[10] Zhang N., Donahue J., Girshick R., Darrell T. Part-based R-CNNs for fine-grained category detection.

[11] Long J., Zhang N., Darrell T. (2014). Do convnets learn correspondence?. *Advances in Neural Information Processing Systems*.

[12] Fischer P., Dosovitskiy A., Brox T. (2014). Descriptor matching with convolutional neural networks: a comparison to SIFT. https://arxiv.org/abs/1405.5769.

[13] Feng Ning F., Delhomme D., LeCun Y., Piano F., Bottou L., Barbano P. E. (2005). Toward automatic phenotyping of developing embryos from videos. *IEEE Transactions on Image Processing*.

[14] Ciresan D. C., Giusti A., Gambardella L. M., Schmidhuber J. (2012). Deep neural networks segment neuronal membranes in electron microscopy images. *Advances in Neural Information Processing Systems*.

[15] Farabet C., Couprie C., Najman L., LeCun Y. (2013). Learning hierarchical features for scene labeling. *IEEE Transactions on Pattern Analysis and Machine Intelligence*.

[16] Pinheiro PH., Collobert R. Recurrent convolutional neural networks for scene labeling.

[17] Hariharan B., Arbeláez P., Girshick R., Malik J. Simultaneous detection and segmentation.

[18] Gupta S., Girshick R., Arbeláez P., Malik J. Learning rich features from RGB-D images for object detection and segmentation.

[19] Ganin Y., Lempitsky V. N4-fields: neural network nearest neighbor fields for image transforms.

[20] Long J., Shelhamer E., Darrell T. (2015). Fully convolutional networks for semantic segmentation. *in Proceedings of the 2015 IEEE Conference on Computer Vision and Pattern Recognition (CVPR)*.

[21] Chavhan G. B., Babyn P. S., Thomas B. (2009). Principles, techniques, and applications of *T*2∗-based MR imaging and its special applications. *Radiographics*.

[22] Arora N., Banerjee A. K., Narasu M. L. (2020). The role of artificial intelligence in tackling COVID-19. *Future Virology*.

[23] Furstenberg R., Kendziora C. A., Stepnowski J. (2008). Stand-off detection of trace explosives via resonant infrared photothermal imaging. *Applied Physics Letters*.

[24] Audebert N., Le Saux B., Lefevre S. (2019). Deep learning for classification of hyperspectral data: a comparative review. *EEE Geoscience and Remote Sensing Magazine*.

[25] Xing C., Ma L., Yang X. (2015). Stacked denoise autoencoder based feature extraction and classification for hyperspectral images. *Journal of Sensors*.

[26] Ramirez Rochac J. F., Zhang N. Feature extraction in hyperspectral imaging using adaptive feature selection approach.

[27] Bahri M., Panagakis Y., Zafeiriou S. (2019). Robust Kronecker component analysis. *IEEE Transactions on Pattern Analysis and Machine Intelligence*.

[28] Jolliffe I. (2005). *Principal Component Analysis*.

[29] Harandi M., Salzmann M., Hartley R. (2018). Dimensionality reduction on SPD manifolds: the emergence of geometry-aware methods. *IEEE Transactions on Pattern Analysis and Machine Intelligence*.

[30] Puggini L., McLoone S. (2017). Forward selection component analysis: algorithms and applications. *IEEE Transactions on Pattern Analysis and Machine Intelligence*.

[31] Zhou J., Kwan C., Ayhan B., Eismann M. T. (2016). A novel cluster kernel RX algorithm for anomaly and change detection using hyperspectral images. *IEEE Transactions on Geoscience and Remote Sensing*.

[32] Olson C. C., Doster T. A novel detection paradigm and its comparison to statistical and kernel-based anomaly detection algorithms for hyperspectral imagery.

[33] Krysko A. V., Awrejcewicz J., Papkova I. V., Szymanowska O., Krysko V. A. (2017). Principal component analysis in the nonlinear dynamics of beams: purification of the signal from noise induced by the nonlinearity of beam vibrations. *Advances in Mathematical Physics*.

[34] Kwan C., Zhou J. (2015). Method for image denoising.

[35] Zhang N., Leatham K. (2019). A neurodynamics-based nonnegative matrix factorization approach based on discrete-time projection neural network. *Journal of Ambient Intelligence and Humanized Computing*.

[36] Ramirez Rochac J. F., Zhang N., Behera P. Design of adaptive feature extraction algorithm based on fuzzy classifier in hyperspectral imagery classification for big data analysis.

[37] Chen LC., Papandreou G., Kokkinos I., Murphy K., AL Y. (2018). DeepLab: semantic image segmentation with deep convolutional nets, atrous convolution, and fully connected CRFs. *IEEE Transactions on Pattern Analysis and Machine Intelligence*.

[38] Aganj I., Harisinghani M. G., Weissleder R., Fischl B. (2018). Unsupervised medical image segmentation based on the local center of mass. *Scientific Reports*.

[39] Chang J., Wang L., Meng G., Xiang S., Pan C. Deep adaptive image clustering.

[40] Krizhevsky A., Sutskever I., Hinton G. E. (2012). Imagenet classification with deep convolutional neural networks. *Advances in Neural Information Processing Systems*.

[41] Micallef N., Seychell D., Bajada C. J. A nested U-net approach for brain tumour segmentation.

[42] Zhou Z., Rahman Siddiquee M. M., Tajbakhsh N., Liang J. U-Net++: a nested U-net architecture for medical image segmentation. *Deep Learning in Medical Image Analysis and Multimodal Learning for Clinical Decision Support, DLMIA 2018, ML-CDS 2018, Lecture Notes in Computer Science*.

[43] Isensee F., Petersen J., Klein A. (2018). nnU-Net: self-adapting framework for u-net-based medical image segmentation. https://arxiv.org/abs/1809.10486.

[44] Li C., Tan Y., Chen W. Attention U-Net++: a nested attention-aware U-net for liver CT image segmentation.

[45] Türk F., Lüy M., Barışçı N. Kidney and renal tumor segmentation using a hybrid V-Net-Based model. *Mathematics*.

[46] Signoroni A., Savardi M., Benini S. (2021). Learning COVID-19 pneumonia severity on a large chest X-ray dataset. *Elsevier, Medical Image Analysis*.

[47] Shi F., Wang J., Shi J. (2021). Review of artificial intelligence techniques in imaging data acquisition, segmentation, and diagnosis for COVID-19. *IEEE Reviews in Biomedical Engineering*.

[48] An J., Zhang X., Zhou H., Jiao L. (2018). Tensor-based low-rank graph with multi-manifold regularization for dimensionality reduction of hyperspectral images. *IEEE Transactions on Geoscience and Remote Sensing*.

[49] Makantasis K., Doulamis A. D., Doulamis N. D., Nikitakis A. (2018). Tensor-based classification models for hyperspectral data analysis. *IEEE Transactions on Geoscience and Remote Sensing*.

[50] Daneshmand P. G., Mehridehnavi A., Rabbani H. (2021). Reconstruction of optical coherence tomography images using mixed low-rank approximation and second order tensor based total variation method. *IEEE Transactions on Medical Imaging*.

[51] Onan A., Korukoğlu S. A feature selection model based on genetic rank aggregation for text sentiment classification. *Journal of Information Science*.

[52] Onan A. Sentiment analysis on Twitter based on ensemble of psychological and linguistic feature sets. *Balkan Journal of Electrical and Computer Engineering*.

[53] Onan A. Ensemble of keyword extraction methods and classifiers in text classification. *Expert Systems with Applications*.

[54] Onan A., Korukoğlu S., Bulut H. A hybrid ensemble pruning approach based on consensus clustering and multi-objective evolutionary algorithm for sentiment classification. *Information Processing & Management*.

[55] Onan A., Korukoğlu S., Bulut H. LDA-based topic modelling in text sentiment classification: an empirical analysis. *International Journal of Linguistics and Computer Applications*.

[56] Onan A. Sentiment analysis on product reviews based on weighted word embeddings and deep neural networks. *Concurrency and Computation: Practice and Experience*.

[57] Onan A. Deep learning based sentiment analysis on product reviews on Twitter.

[58] Onan A. Sentiment analysis on massive open online course evaluations: a text mining and deep learning approach. *Computer Applications in Engineering Education*.

[59] Onan A. Topic-enriched word embeddings for sarcasm identification. *Software Engineering Methods in Intelligent Algorithms. CSOC 2019. Advances in Intelligent Systems and Computing*.

[60] Onan A. (2017). Hybrid supervised clustering based ensemble scheme for text classification. *Kybernetes*.

[61] Onan A., Toçoğlu M. A. A term weighted neural language model and stacked bidirectional LSTM based framework for sarcasm identification. *IEEE Access*.

[62] Onan A. (2016). An ensemble scheme based on language function analysis and feature engineering for text genre classification. *Journal of Information Science*.

[63] Sabale S. P., Jadhav C. R. Hyperspectral image classification methods in remote sensing—a review.

[64] Ramirez Rochac J. F., Zhang N. Reference clusters based feature extraction approach for mixed spectral signatures with dimensionality disparity.

[65] Ramirez Rochac J. F., Zhang N., Xiong J., Zhong J., Oladunni T. Data augmentation for mixed spectral signatures coupled with convolutional neural networks.

